RETRACTED

# Effects of Different Intervention Methods on Intestinal Cleanliness in Children Undergoing Colonoscopy

**DOI:** 10.1155/2022/1898610

**Published:** 2022-04-16

**Authors:** Yirong Yang, Yuan Xiao, Li Zhang, Jiajia Lv, Qiyun Huang

**Affiliations:** ^1^Department of Nursing, Ruijin Hospital Affiliated to Shanghai Jiaotong University School of Medicine, Shanghai 200025, China; ^2^Department of Pediatrics, Ruijin Hospital Affiliated to Shanghai Jiaotong University School of Medicine, Shanghai 200025, China; ^3^Department of Radiotherapy, Ruijin Hospital Affiliated to Shanghai Jiaotong University School of Medicine, Shanghai 200025, China

## Abstract

**Objective:**

To explore the effects of different intervention methods on intestinal cleanliness in children undergoing colonoscopy.

**Methods:**

61 children who underwent colonoscopy in our hospital from May 2020 to May 2021 were randomly divided into group A (*n* = 21), group B (*n* = 30), and group C (*n* = 10). The children in the three groups were intervened in different ways before the colonoscopy. Group A received a long-handled Kaiselu +1 cathartic intervention, while group B received a long-handled Kaiselu +2 cathartic intervention, and group C received an enema plus one cathartic intervention. The patients in the three groups were given the same diet before the examination until the examination was completed. The time-related indexes, cleanliness, adverse reactions, tolerance, and adaptability of the three groups under different dietary interventions and cleaning methods were evaluated.

**Results:**

The first defecation time in group C was lower than that in group A and group B, the hospital stay was longer than that in group A and group B (*p* > 0.05), and the colonoscopy time in group C was shorter than that in group A and group B (*p* < 0.05). The BBPS score of group C was (2.10 ± 0.32), which was significantly higher than that of group A (1.16 ± 0.19) and group B (1.77 ± 0.18) (*p* < 0.05). The BBPS scores of children with liquid food in the three groups were significantly higher than those of common food, and the BBPS scores of liquid food and common food in group C were significantly higher than those in group A and group B (*p* < 0.05). The incidence of adverse reactions in group C was 20.00%, which was significantly lower than 33.33% in group A and 23.33% in group B (*p* < 0.05). The proportion of grade I in group C was 50.00%, which was significantly higher than 38.10% in group A and 43.33% in group B (*p* < 0.05).

**Conclusion:**

Children undergoing colonoscopy take preintestinal preparation under different diets and intervention methods. The cleanliness of liquid food and enema + one-time laxative one day before colonoscopy is the best, which can significantly reduce adverse reactions and increase the acceptability and adaptability of children. It is worthy of clinical application.

RETRACTED

## 1. Introduction

As one of the clinical fiber endoscopes, colonoscopy can observe the internal conditions of the rectum, colon, cecum, and part of the small intestine through anal reverse insertion. The lesions and degree of the digestive system can be clearly understood by using an objective lens and a light image conversion system to assist in clinical surgical examination and operation [1, 2]. Colonoscopy has been used for pediatric digestive tests since the 1980s. As the main examination method for the diagnosis of colorectal diseases in children, its disease detection rate and safety are high, and it is widely used in pediatrics [3]. Whether colonoscopy can be carried out smoothly depends mainly on intestinal preparation. High-quality intestinal preparation can not only clear the observed lesion location and degree, improve the disease detection rate and the success rate of endoscopic treatment, but also shorten the examination time. At the same time, it is convenient for medical staff to check the operation and relieve patients' discomfort [4, 5]. During clinical colonoscopy for children, the examination is often performed under general anesthesia, considering the acceptance degree, physical dosage, and tolerance of children. Intestinal examination preparation should be arranged according to child's age, physical condition, clinical symptoms, digestive status, and examination willingness [6]. At present, there are many preparation programs, among which physiological saline enema, oral magnesium sulfate, or mannitol are important drugs for adults to clean the intestine before examination. However, it may cause adverse reactions such as hypoglycemia, and the cleaning effect is not good. Therefore, it is necessary to further find a safer, feasible, and cleaner plan for the intestinal preparation of children [7, 8]. Casserole long stem uses hypertonic reactions caused by glycerin or sorbitol to soften metabolites and stimulate intestinal wall reflexes to cause defecation behavior, which has limited stimulation to the body and is often applied in constipation and intestinal preparation with minor adverse reactions [9, 10]. In this study, children undergoing colonoscopy were treated with different intestinal prepreparation interventions since May 2020, aiming to explore the effects of different interventions on intestinal cleanliness and comfort of general diet and liquid food. The report is as further discussed in this study.

## 2. Data and Methods

### 2.1. General Information

In this study, 61 children who underwent colonoscopy in our hospital from May 2020 to May 2021 were selected as the subjects and randomly divided into group A (*n* = 21), group B (*n* = 30), and group C (*n* = 10) according to the time of admission. There were 9 males and 12 females in group A with an average age of 11 ± 1.2 months, including 2 abdominal distension, 2 diarrhea, 2 constipation, 1 mucus, and no fistula. In group B, there were 14 males and 16 females, with an average age of 9.2 ± 0.8 months, including 1 case of abdominal distension, 12 cases of diarrhea, 2 cases of constipation, 1 case of mucus, and no fistula. In group C, there were 7 males and 3 females, with an average age of 8.4 ± 0.6 months, including 2 abdominal distension, 3 diarrhea, 1 mucus, no fistula, or constipation. There was no significant difference in baseline data between the three groups (*p* > 0.05), indicating comparability. Before colonoscopy, three groups of children were given different interventions: group A was given carcerol long-stalk +1 time of laxative intervention, group B was given carcerol long-stalk +2 times of laxative intervention, and group C was given enema +1 time of laxative intervention. All patients in the three groups were given the same diet before the examination until the examination was completed. This study was approved by the hospital medical committee.

RETRACTED

### 2.2. Inclusion and Exclusion Criteria

The inclusion criteria were as follows: (1) in line with the diagnostic indication criteria in Expert Consensus on Standardized Operation of Gastroscopy and Colonoscopy for Children in China [11]; (2) the colonoscopy was performed for the first time, and the colonoscopy criteria were met; (3) aged from 3 to 18; (4) clinical manifestations include lower gastrointestinal bleeding, abdominal pain, diarrhea, anemia, perianal lesions, and lower gastrointestinal diseases; (5) no cognitive impairment, mental system diseases, and so on; and (6) complete clinical data; study subjects, family members or legal guardians, were informed of the contents of the project and signed informed consent.

The exclusion criteria were as follows: (1) patients with serious dysfunction of heart, liver, kidney and blood vessels; (2) with intestinal obstruction, gastrointestinal bleeding or perforation, intestinal infection, toxic enteritis, and intestinal volvulus; (3) complicated with peritonitis, abdominal mucosa, megacolon crisis, and abdominal malignant tumor; (4) patients with hypertension, hyperglycemia, and other chronic diseases; (5) With moderate or severe diarrhea and constipation; (6) with coagulation disorder, allergic to the study drugs or have a history of severe allergy; and (7) poor compliance, do not cooperate with visitors.

RETRACTED

### 2.3. Research Methods

Preenteral preparation: after admission, all children were given psychological education, explaining the examination items and telling their relatives to soothe their anxiety. The history of allergy, surgery, disease, and medication was filled in, and the specific physical symptoms and basic information were explained. A blood routine, a urine routine, and a cardiohepatic examination were performed. The diet, medication, time arrangement, and matters needing attention during the preparation period were informed. The number of defecations, character, and physiological reactions were observed during the preparation period. According to the physical condition and tolerance of children, all patients in the three groups ate as recommended the day before the examination. In group A, there was 1 case of liquid food, 10 cases of semiliquid food, and 10 cases of general food. In group B, there were 3 cases of liquid diet, 8 cases of semiliquid diet, and 19 cases of general diet. In group C, there were 2 cases of liquid diet, 3 cases of semiliquid diet, and 5 cases of general diet. In order to prevent hypoglycemia, a supplement glucose electrolyte solution was given before the examination. At the same time, fasting was recommended for 4h to 6h before liquid food examinations and 8h before general food examinations according to different types of diet.

According to the Intestinal Preparation Guidelines related to the Diagnosis and Treatment of Digestive Endoscopy in China [12], the dosage requirements of Kaiselu, compound polyethylene glycol electrolyte powder (Shutaiqing (Beijing) Biopharmaceutical Co., Ltd.; State Drug Approval H20040034), and enema for all children were based on their physique, weight, and degree of disease. One day before the examination, after dietary management, all patients were given compound polyethylene glycol electrolyte powder orally, 300g in 3000 mL, and it was taken completely internally for 1h. Among them, patients in group B received 80 mL/kg polyglycol electrolyte again at 8 : 00 a.m. on the day of examination. Patients in group A and group B were treated with long-handled Kaiselu intervention. All the glycerin in Kaiselu (20 ml) was inhaled into a syringe (without a needle), a part of the scalp needle was inserted and paraffin oil was applied, and the needle was slowly inserted into the child's anus to the scalp, and the drug solution was slowly injected into the rectum for 10 to 20 minutes before defecation. Group C was given a normal saline enema and a glycerin enema after admission. Children under 3 years old were given 250 ml of warn water. At the age of 4–6 years old, 550 ml of warn water given. From 6 to 9 years old, 800 ml of warn water was given. Aged 10 years and above, 1100 ml of warn water was given. During the guidance of the prone position, it was kept longer.

RETRACTED

### 2.4. Observation Indicators

Time-related indicators were evaluated, including time of initial defecation, colonoscopy time, and length of hospital stay, wherein colonoscopy time was the time from colonoscopy insertion to complete withdrawal. (2) Evaluation of intestinal cleanliness after different intervention methods: the Boston Bowel Preparation Scale [13] (BBPS) was used to measure the quality of bowel preparation in the three groups, which divides the colon into three parts. They were the right colon (ileocecal colon, ascending colon), the middle colon (transverse colon, descending colon), and the left colon (sigmoid colon, rectum), with a total of 3 points for each colon and a total of 9 points. The higher the score, the better the cleaning effect. (3) To evaluate the intestinal cleanliness of different diets; (4) the incidence of adverse reactions in the three groups was evaluated, including nausea, vomiting, abdominal distention, abdominal pain, cold sweat, palpitation, and dizziness; (5) the tolerance and comfort level of the children in the three groups were evaluated. After colonoscopy, questionnaire survey was conducted to evaluate their comfort level and tolerance. And ask if you would like to have another colon examination or preparation.

### 2.5. Clinical Evaluation Criteria

Performed and recorded by the same experienced endoscopic surgeon, intestinal cleanliness was assessed by the double-blind method.

The scoring standard for the segmented cleanliness of the intestinal tract was as follows [14]: the intestinal tract was poorly cleaned, the intestinal lumen was filled with a large amount of feces and feces residue, and no mucous membrane was found, so the endoscopic observation was not possible, and it was judged as 0. Intestinal cleanliness is poor, a large number of feces and feces residue can be seen in the intestinal lumen, and some mucous membranes can be seen. Experienced patients can be forced into the microscope and observation, and it is judged as 1 point. Intestinal cleanliness was fair, a small amount of feces and fecal residue remained in the intestinal lumen, and mucous membrane could be seen. There was no obstruction in endoscopic and observation, and the field of vision was still clear, which was judged as 2 points. The intestinal tract was well cleaned, no feces or feces residue was found in the intestinal lumen, the mucous membrane was clearly visible, and the field of vision was good, which had no influence on the endoscopy and observation. It was judged as 3 points.

RETRACTED

Overall intestinal cleanliness scoring standard [15]: the total score is less than 5 points or the score in any section is less than 2 points, which indicates that the intestinal fecal and fecal residue accumulation during colonoscopy is serious and the examination cannot be carried out smoothly. The total score of 6–7 was judged as good intestinal cleanliness, indicating that the residual feces and fecal residue in the intestinal tract during colonoscopy would not affect the observation and treatment under colonoscopy. Those with a total score of 8–9 were judged to have excellent intestinal cleanliness, indicating that there was no feces and fecal residue in the intestine during colonoscopy, and the intestine was fully prepared.

Tolerance evaluation criteria [16]: i degree no obvious discomfort, complete tolerance, complete acceptance of second colonoscopy, and preparation. Degree ii mild discomfort, tolerable, but acceptable for a second colonoscopy and preparation. Grade iii was moderate/severe discomfort, totally intolerable, and the second colonoscopy was refused and prepared.

### 2.6. Statistical Treatment

The data were processed by SPSS 24.00 statistical software. The measurement data were expressed as *X* ± *S*, and comparison between groups was performed by the *T* test. The counting data were expressed as case number (*n*) and percentage (%). The *χ*2 test was used for comparison between groups, and *p* < 0.05 indicated statistically significant differences.

## 3. Results

### 3.1. Comparison of Time-Related Indicators

The results showed that the time of initial defecation in group C was shorter than that in groups A and B, and the length of hospital stay was longer than that in groups A and B, with no statistical significance (*p* > 0.05). The colonoscopy time of group C was shorter than that of group A and group B. The difference was statistically significant (*p* < 0.05), as shown in Table 1.

### 3.2. Comparison of Intestinal Cleanliness with Different Intervention Methods

The results showed that the BBPS score of group C (2.10 ± 0.32) was significantly higher than that of group A (1.16 ± 0.19) and group B (1.77 ± 0.18). The difference was statistically significant (*p* < 0.05), as shown in Figure 1.

### 3.3. Comparison of Intestinal Cleanliness between Different Diets

The results showed that the BBPS score of liquid food in three groups was significantly higher than that of general food, and the difference was statistically significant (*p* < 0.05). The BBPS scores of liquid diet and general diet in group C were significantly higher than those in group A and group B. The difference was statistically significant (*p* < 0.05), as shown in Table 2.

RETRACTED

### 3.4. Comparison of Incidence of Adverse Reactions

The results showed that the incidence of adverse reaction in group C (20.00%) was significantly lower than that in group A (33.33%) and group B (23.33%). The difference was statistically significant (*p* < 0.05), as shown in Table 3.

### 3.5. Comparison of Tolerance and Comfort

The results showed that the proportion of i degree in group C (50.00%) was significantly higher than that in group A (38.10%) and group B (43.33%). The difference was statistically significant (*p* < 0.05), as shown in Table 4.

## 4. Discussion

With the change of people's health consciousness and eating habits, the examination of the upper and lower digestive tract has been paid more and more attention. As a major examination device, colonoscopy can accurately detect the location, type, and degree of lesions in the colon with significant safety and feasibility [17]. The accuracy and quality of colonoscopy largely depend on the cleanliness of intestinal pre-preparation. Excellent cleanliness can smoothly insert the colonoscopy, observe the mucosa and pathological tissues, and improve the detection rate and treatment success rate of intestinal diseases [18]. Intestinal cleanliness quality is closely related to many factors, including diet before examination, dosage and frequency of laxative, patient psychology, and disease status. At present, most studies at home and abroad focus on adult disease types, laxative selection and dosage, diet, and other aspects. Most scholars believe that liquid or semiliquid food should be eaten one day before the examination, and fasting should be required for 4 to 6 hours before the examination. Biopsy or treatment is not suitable for such patients, and a large number of samples are required for verification. However, domestic studies on the intestinal preparation of children are limited, especially in dietary control [19, 20]. Due to the gastrointestinal function development and dietary habits of children, the probability of colonoscopy is increasing year by year, and the demand for pediatric gastrointestinal preparation is increasing [21]. In this study, children who underwent colonoscopy were treated with different dietary controls and cathartic interventions, respectively, to observe the cleanliness, tolerance, and adaptability of intestinal preparation in each group.

There are many kinds of drugs for intestinal preparation before colonoscopy, and their combinations and uses are different. Due to the weak gastrointestinal function of children, medication and dose need to be improved. Shan *J* et al. [22] separately administered polyethylene glycol electrolytes to patients undergoing morning colonoscopy for intestinal prepreparation with a separate dose and a single dose, and BBPS scores in the separate dose group were significantly higher than those in the single dose group, showing more significant tolerance and satisfaction. Gimeno-Garcia AZ et al. [23] believed that a low-residue diet was more conducive to improving intestinal cleanliness in patients undergoing colonoscopy during intestinal prepreparation, especially the effect of liquid or semiliquid food intake one day before the examination was more significant. The results of this study showed that the colonoscopy time of group C was shorter than that of group A and group B; the BBPS score of group C (2.10 ± 0.32) was significantly higher than that of group A (1.16 ± 0.19) and group B (1.77 ± 0.18). The BBPS score of liquid diet was significantly higher than that of general diet in the three groups, and the BBPS score of liquid diet and general diet in group C was significantly higher than that in group A and group B. Similar to the study of Shan *J* and Gimeno-Garcia AZ, it indicated that taking liquid food, enema, and one laxative one day before colonoscopy had the most significant cleaning effect. Semifluid diet in intestinal preparation can drain the colon in a short time and does not cause changes in colonic protein, water electrolyte, and mucosa. In addition, it is necessary to meet the physiological needs of children, improve the cleanliness of the colon, and reduce the impact on colonoscopy. Enema combined with polyethylene glycol electrolyte can increase the osmotic pressure in the colon, have the advantages of being rapid and thorough, and reduce the colon empty time. At the same time, it will not cause electrolyte disorder in the field, reduce the intestinal examination time and discomfort of children, making it more suitable for children with intestinal fragility.

RETRACTED

During intestinal preparation, different patients may experience adverse reactions such as nausea, abdominal distension, and cold sweat due to different physical signs, gastrointestinal function, and tolerance degree. In addition, due to the metabolic imbalance of the body itself, it will aggravate gastrointestinal dysfunction and affect the detection rate and treatment rate of microscopic lesions by colonoscopy. Chen *E* et al. [24] used low-residue food and no-residue food, respectively, for adenocarcinoma patients undergoing colon cancer examinations. The results showed that there was no significant difference in cleanliness between the two diets. The tolerance degree and fitness degree of patients with a low-residue diet were higher than those with a clear liquid diet, and the hunger of patients was reduced. Yokoi A et al. [25] applied olive oil enema for children with severe chronic constipation, and the results showed that olive oil had a significant lubrication effect and could treat most children with good results, with ideal tolerance effect and adaptability. The results showed that the incidence of adverse reactions in group C was significantly lower than that in group A and group B. The proportion of degree i in group C was significantly higher than that in group A and group B. Similar to the study of Chen *E* and Yokoi A, it indicated that children undergoing colonoscopy had a lower risk of adverse reactions and a higher tolerance and adaptability by eating dreg-free food, enema, and one laxative for intestinal preparation one day before the colonoscopy. As a commonly used laxative, Kaiselu is passed into the rectum through glycerin or sorbitol to soften the stool and stimulate the intestinal physiology to cause a defecation reaction. Glycerin will accompany lubrication, making it more conducive to defecation. However, carcerol can cause swelling and pain in the perianal mucosa in children and even stimulate the rectal mucosa, causing discomfort in children. Through warm water or physiological saline enema to promote physical absorption of water in the large intestine and maintain the body water and electrolyte balance. At the same time, can use pressure or chemical stimulation to promote spontaneous defecation and improve the coordination and tolerance of children.

## 5. Conclusion

In conclusion, children undergoing colonoscopy can eat liquid or semiliquid food 1d before the examination and take one enema and laxative bowel preparation to achieve ideal intestinal cleanliness, reduce the incidence of adverse reactions, improve the tolerance and adaptability of children, and provide a good intestinal environment for clinical examination and treatment. However, the following problems still exist in this study: the sample size is limited, so it is necessary to expand the sample size to explore its universality. The follow-up time is short, so it is necessary to observe the gastrointestinal injuries of children for a long time and adopt appropriate laxatives. The scope of the study is one-sided, and the influence of other factors of intestinal cleanliness on the experimental results should be discussed.

## Figures and Tables

**Figure 1:** Comparison of BBPS scores by different intervention methods (note, compared with group (C) ^*∗*^*p* < 0.05).

**Figure 2:** Comparison of BBPS scores of different dietary patterns (left: group A; middle: group B; right: group C; note: compared with liquid diet, ^*∗*^*p* < 0.05; compared with group (C) (^*∗*^*p* < 0.05).

RETRACTED

**Table 1:** Comparison of time related indicators ($\bar{x}$ ±*s*).

Group	Group A	Group B	Group C	F	*p*
	(*n* = 21)	(*n* = 30)	(*n* = 10)		
Time of first defecation (min)	8.32 ± 1.92	8.25 ± 1.89	8.03 ± 1.97	0.253	0.316
Colonoscopy time (min)	21.79 ± 8.46	18.65 ± 7.24	14.09 ± 6.03	2.420	0.025
Length of hospital stay (D)	3.54 ± 0.68	3.94 ± 0.72	4.23 ± 0.79	4.071	0.102

**Table 2:** Comparison of BBPS scores by different dietary patterns (*χ*±*s*).

Group	Group A	Group B	Group C
	(*n* = 21)	(*n* = 30)	(*n* = 10)
Liquid diets	1.22 ± 0.32^#^	1.91 ± 0.34^#^	2.20 ± 0.37
Ordinary food	1.08 ± 0.19^*∗*^^#^	1.67 ± 0.23^*∗*^^#^	2.00 ± 0.55^*∗*^

Note: compared with liquid diet, ^*∗*^*p* < 0.05. Compared with group C, #*p* < 0.05, as shown as Figure 2.

**Table 3:** Comparison of adverse reaction rate (cases, %).

Group	Group A	Group B	Group C	F	*p*
	(*n* = 21)	(*n* = 30)	(*n* = 10)		
Nausea	1 (4.76)	2 (6.67)	0 (0.00)	—	—
Vomiting	0 (0.00)	1 (3.33)	1 (10.00)	—	—
Abdominal distension	2 (9.52)	2 (6.67)	0 (0.00)	—	—
Abdominal pain	2 (9.52)	1 (3.33)	1 (10.00)	—	—
Cold sweat	1 (4.76)	0 (0.00)	0 (0.00)	—	—
Heart palpitations	0 (0.00)	1 (3.33)	0 (0.00)	—	—
Dizzy	1 (4.76)	0 (0.00)	0 (0.00)	—	—
Incidence of adverse reactions	33.33%	23.33%	20.00%	1.214	0.001

**Table 4:** Comparison of tolerance and comfort (cases, %).

Group	Group A	Group B	Group C
	(*n* = 21)	(*n* = 30)	(*n* = 10)
I	8 (38.10)	13 (43.33)	5 (50.00)
II	7 (33.33)	10 (33.33)	3 (30.00)
III	6 (28.57)	7 (23.33)	2 (20.00)

## Data Availability

The data used to support the findings of this study are available from the corresponding author upon request.
